# An Early Warning Risk and Control Model for Manpower Capital Investment Using Data Warehousing and Computational Intelligence

**DOI:** 10.1155/2022/7624135

**Published:** 2022-03-24

**Authors:** Yang Liu, Zongyu Wang

**Affiliations:** ^1^School of Economics and Management, Harbin University of Science and Technology, Harbin, Heilongjiang 150080, China; ^2^School of Electronics and Information Engineering, Heilongjiang University of Science and Technology, Harbin, Heilongjiang 150022, China

## Abstract

Human capital plays an important role in the development of enterprises. Investing in human capital is the main focus of enterprises to improve personnel quality and enhance their core competitiveness. With the development of market economy, the function of human resource market allocation has been improved and the mobility of enterprise human resources has been enhanced leading to the increase in investment risk of enterprise human capital. Enterprise human capital investment risk has a negative impact on enterprises, reduces the income of enterprises' human capital investment, and affects their growth. Hence, enterprises need to avoid the risk of human capital investment or minimize the negative impact of risk. Using the data warehouse and computational intelligence, this paper constructs the early warning and control model for human capital investment risk and analyzes the existing approaches during the recruitment process and training, investment, and production, among enterprises. Finally, this paper proposes the corresponding control method according to the model inspiration.

## 1. Introduction

In the trend of economic globalization and international economic integration, the competition among countries in the world is becoming more and more intense. With the advent of the knowledge economy, knowledge has become the basis of development [1]. Because the carrier of knowledge is the individual in the enterprise, the basis for the survival and development of modern enterprises is rooted in the manpower capital of enterprises. Advanced science and technology needs a strong economic foundation for support. Enterprises are the basic unit of the national economy. The operation status of enterprises affects the national economic strength, so the state should pay attention to the development of enterprises [2]. Manpower capital plays a very important role in enterprise development. Manpower capital investment is the main means for enterprises to improve personnel quality and enhance their core competitiveness [3]. The development of the market economy improves the function of human resources market allocation, and the liquidity of enterprise human resources is enhanced, resulting in the increase of enterprise manpower capital investment risk [4]. Enterprise manpower capital investment management risk refers to the uncertainty of income and the possibility of loss caused by the enterprise's unclear understanding of the attributes of manpower capital in various manpower capital investments, such as self-interest, initiative, personal property right attribute, and comprehensive matching [5]. The advantage of enterprise manpower capital is equal to the core competitiveness of enterprises. In this development trend, enterprises, as economic organizations with the goal of maximizing profits, have taken manpower capital investment as an important strategy for enterprise survival and development [6].

Like other investments, manpower capital investment also has risks and some special attributes of manpower capital determine that the investment in manpower capital is different from that in other factors [7]. The loss of enterprise manpower capital causes the reduction or loss of manpower capital investment income, brings investment risks to enterprises, reduces the enthusiasm of enterprises for manpower capital investment, and is very unfavorable to the long-term development of enterprises [8]. The dependence, heterogeneity, and dynamics of manpower capital make the investment income uncertain, the forms are diversified, and the payback period of investment is long, which exacerbates the risk of manpower capital investment [9]. Like other investments, manpower capital investment has great risk. Manpower capital investment risk cannot be ignored by enterprises. How to treat manpower capital investment rationally and make manpower capital investment decisions carefully, so as to reduce or avoid manpower capital investment risk and maximize manpower capital investment income, has become an important research topic [10]. Data warehouse technology provides enterprises with solutions to analyze and mine a large amount of historical data accumulated within the enterprise and possible external information and extract valuable information from it, so as to help managers analyze business conditions [11]. Based on data warehouse technology, this paper constructs a risk early warning and control model of manpower capital investment, analyzes the game in the process of recruitment, training, investment, and production, and gives the corresponding treatment scheme according to the enlightenment of the model. Finally, based on the analysis of game theory, this paper makes a supplementary summary and puts forward the preventive countermeasures against the risk of enterprise manpower capital investment.

The proportion of the tertiary industry in the national economy is increasing. Like some high-tech industries and service industries, the contribution rate of their manpower capital to enterprise development accounts for the vast majority [12]. Its manpower capital value also determines most of the value of the enterprise and also determines the future value of the enterprise. The risk of enterprise manpower capital investment will bring many negative effects to the enterprise, reduce the income of enterprise manpower capital investment, and affect the growth of the enterprise [13]. Therefore, enterprises should try to avoid the risk of manpower capital investment or minimize the negative impact of risk on enterprises. The development prospect and future destiny of the enterprise are controlled by the talents of the enterprise, who have rich management experience, profound knowledge, exquisite skills, and active innovative thinking [14]. Their economic behavior directly determines the fate of enterprises and the economic strength of the country. The special attributes of manpower capital, such as heterogeneity and dependence, determine that the risk of manpower capital investment is personalized [15]. Using data warehouse technology to strengthen enterprise risk management plays an important role in modern enterprise management. Enterprises can effectively reduce and eliminate human operation risks and enhance customer maintenance ability by establishing an efficient data warehouse, centralizing decentralized business systems, unifying and solidifying business processing processes, and standardizing management means.

Firstly, this paper discusses the basic concepts of human capital investment and data warehouse and, on this basis, puts forward the early warning and control model of human capital investment risk based on data warehouse technology. Then, in Section 4 of the article, the simulation results of the algorithm are analyzed, the effectiveness of the early warning model of human capital investment risk is verified, and the risk control strategy is put forward.

## 2. Related Work

In the process of its development and perfection, manpower capital theory is increasingly accepted by people. People began to realize the importance of manpower capital to social progress and economic development and actively invested in manpower capital, hoping to get rich benefits from it. Literature [16] holds that investment in education is unsafe, investment in higher education bears considerable risks, and this kind of investment is not easy to change. Literature [17] points out that the causes of manpower capital investment risk can be analyzed from three levels: external environment government, internal environment enterprises, and individuals. Literature [18] holds that the root of the moral hazard of manpower capital lies in the inconsistency of material interests between principal and agent, information asymmetry, and environmental uncertainty. Literature [19] pointed out that modern portfolio theory should be used to spread the risk of manpower capital investment. Literature [20] holds that, unlike portfolio investment, the risk of manpower capital investment is often personalized and manpower capital is an illiquid asset. It established the pricing model of manpower capital and brought nonlinear assumptions, labor supply, and risk financial assets into the model to achieve the optimal investment model of manpower capital. Literature [21] holds that the key to preventing and controlling the artificial risk of investors is to improve the internal management of enterprises, establish the incentive and restraint mechanism of manpower capital, and eliminate the inducing factors of this risk beforehand. Literature [22] pointed out that more investment in universal manpower capital from the individual point of view can better avoid risks. Literature [23] shows that education can help a person avoid low-income or low-paid jobs to reduce the risk of unemployment, so we should increase investment in manpower capital.

In this paper, the risk of manpower capital investment is identified from the perspective of management, and the early warning and control model of manpower capital investment risk is constructed, so that enterprises can understand the causes and evaluation methods of risk, find out the changing trend of risk, and find preventive measures to reduce the risk of manpower capital investment.

## 3. Materials and Methods

### 3.1. Manpower Capital Investment Theory

Human resource planning refers to the determination of the quantity and quality of human resources needed for enterprise development in a certain period of time in the future according to the requirements of enterprise development strategy. The acquisition of these human resources may come from within the enterprise, or from the society and campus. For enterprises, this can also be regarded as an investment, because there will also be an investment in human and financial resources when making plans [24]. There are usually specific skills training, etiquette or moral training for all employees, and management knowledge training for managers. Through the assessment and evaluation of employees' daily behaviors and work results, we can find the advantages and disadvantages of employees at work. Good salary and welfare benefits can motivate employees to work better and promote the effective play of manpower capital. This investment method is an important means to improve the utilization rate of manpower capital and employee relationship management.

### 3.2. Data Warehouse

When an enterprise carries out the same manpower capital investment plan, if the investment objects are different employees, the investment gains and effects will be different. Some employees of enterprises may agree with this kind of training method in their hearts, and it is easier to accept and absorb this kind of investment content and investment method when training. On the contrary, other employees may have resistance. These reasons are all factors that enterprises need to consider when investing in manpower capital. The value of manpower capital management is reflected in the daily business operation, namely, business analysis and decision-making. The data warehouse serves the business, that is, provides support for decision-making. From the enterprise's point of view, an investment plan may best meet the enterprise development strategy and current investment needs, but as the recipient of investment content, enterprise employees may be influenced by personal preferences and emotions, may think that they do not meet their own wishes, or may have little improvement on their own growth, and enterprises will not get the best investment status if employees do not cooperate or actively try to absorb it [25]. From the technical point of view, a data warehouse is a database system that meets the basic model of a data storage center. From the user's point of view, it reorganizes the existing data and the data to be generated and effectively improves the consistency, integrity, integration, and system performance of the data, so as to better serve the user's query, analysis, decision support, and data mining.

In order to accurately understand the customer's behavior to support the marketing and risk departments, we must be able to integrate and collect massive customer information, so as to analyze and obtain accurate customer characteristics, especially risk characteristics. The technical core of realizing this kind of manpower capital management is a data warehouse. The storage structure design of the data warehouse system is shown in Figure 1.

### 3.3. Early Warning and Control Model of Manpower Capital Investment Risk

As an entity, enterprise employees who are the objects of manpower capital investment have a life cycle and an economic life cycle. With the increase in people's age, the production and transformation efficiency of manpower capital will decrease. With the shortening of the economic life cycle, the sustainable income that enterprises can obtain from enterprise employees will also decrease. Moreover, after the investment of enterprise manpower capital is completed, the ability of manpower capital is also related to the enterprise environment, incentive system, and other influencing factors. At present, there are many definitions of data warehouse, which makes it difficult to make a clear explanation strictly. Enterprise manpower capital investment risk early warning has the given functions for enterprise manpower capital investment decision-making and project implementation, as shown in Figure 2.

The uncertainty of the investment income of enterprise manpower capital refers to the possibility that the investment income obtained after a period of transformation of enterprise investment is lower than the expected investment income. The possibility that the loss of enterprise manpower capital investment occurs refers to the possibility that the investment income obtained after the joint efforts of employees and enterprises is lower than the investment cost. The two can be represented visually by mathematical formulas, respectively, as follows:

(1) $$\begin{array}{c} D_{i}=a+\sum_{j=1}^{n}b_{j}p_{j}+r_{i}Y+u,\\ D_{i}=a+\sum_{j=1}^{n}b_{j}\ln\left(p_{j}\right)+r_{i}\ln\left(Y\right)+u. \end{array}$$

Among them, a is the profit period of manpower capital investment and *b* is the cost period of manpower capital investment. *D*_*i*_ is the actual income of manpower capital investment, *p* is the expected income of manpower capital investment, and Y is the cost of manpower capital investment.

Technically, the data warehouse is a database, but it is different from the database of a daily business system. The goal of building a data warehouse system is to build a data storage center that can integrate various departments and sources [26]. It regards the information distributed in different departments as the important information resources of the data warehouse, and through convenient, flexible, efficient, and automatic data extraction, conversion, assembly, and cutting tools, it converts, cleans, and integrates the required data, transfers the correct, consistent, and complete data to the data warehouse system, and effectively manages the data warehouse. Whether the incentive system, welfare, and benefits of the enterprise are reasonable and whether the working environment and working atmosphere of the enterprise are harmonious, all affect the creativity of the employees' manpower capital, thus affecting the ultimate income of the enterprise. The uncertainty of investment objects is one of the reasons for the risk of manpower capital investment.

Assume that the manpower capital investment risk of an enterprise has *n* mutually incompatible states, and its initial state is as follows:

(2) $$\begin{array}{c} S^{\left(0\right)}=\left[S_{1}^{\left(0\right)},S_{2}^{\left(0\right)},\cdots ,S_{n}^{\left(0\right)}\right]. \end{array}$$

Among them, *S*_*t*_^(0)^(*t*=1,2,3, ⋯, *n*) is the initial probability of being in state *t*; if the state probability of being in stage *i* after the k-step transition is *S*_*i*_^(*k*)^(*t*=1,2,3, ⋯, *n*), we know the following:

(3) $$\begin{array}{c} S_{j}^{\left(k+1\right)}=\sum S_{i}^{\left(k\right)}\times P_{ij}\left(j=1,2,\cdots ,n\right). \end{array}$$

This is converted into the following matrix form:

(4) $$\begin{array}{c} S^{\left(k+1\right)}=S^{k}\times P. \end{array}$$

It can be derived from the following:

(5) $$\begin{array}{c} S^{\left(k+1\right)}=S^{k}\times P=S^{\left(0\right)}\times P^{\left(k+1\right)}. \end{array}$$

Enterprise manpower capital investment risk early warning is to monitor unsafe behaviors in enterprise manpower capital investment activities. Once any deviation from the investment plan or other abnormalities is found, one should analyze these abnormal behaviors immediately, find out the influencing factors in the investment process, and diagnose the “contribution” of these influencing factors to the possibility of risk occurrence. According to the investment plan, the enterprise arranges the investment contents and means. However, due to the long investment time, some unexpected things may happen in the middle and it is necessary to make some adjustments to the previous plan. Risk identification is the basis of risk early warning of manpower capital investment in the whole enterprise. Without risk identification, it is impossible to carry out scientific risk early warning activities. Enterprise manpower capital investment risk identification is to analyze and study the various influencing factors that may cause risks, judge the possibility of all kinds of risks, and summarize all kinds of manpower capital investment risks that enterprises may face before the risks occur. Because of the long-term nature of enterprise manpower capital investment, there are some uncertain factors. In the investment process, especially in the training process, trainers and trainees should be properly supervised to ensure the efficiency of investment.

Sort the hierarchical list, check the consistency of the pairwise comparison matrix, and revise it if necessary to achieve the correctable consistency. The square root method is used to calculate the approximate value of index weight.

We calculate the product of each element in each row of the judgment matrix:

(6) $$\begin{array}{c} P_{d}=N_{i}v_{i}\left(\frac{M_{i}v_{i}^{2}}{2}+Zeu\left(t\right)\right). \end{array}$$

We calculate the power root of the feature quantity:

(7) $$\begin{array}{c} E_{c}=2\sqrt{\frac{ZeN_{i}}{\varepsilon_{0}}\left(\sqrt{u\left(t\right)U_{0}+U_{0}^{2}}-U_{0}\right)}. \end{array}$$

We normalize the vector:

(8) $$\begin{array}{c} Y_{j}\left(t\right)=\phi \left(\sum_{i=1}^{n}w_{ji}x_{i}-\theta_{j}\right). \end{array}$$

The vector *n* is the weight vector to be sought. We find the maximum eigenvalue of the matrix:

(9) $$\begin{array}{c} o_{j}\left(t\right)=f\left(\left[\sum_{i=1}^{n}w_{ij}x_{i}\left(t-\tau_{ij}\right)\right]-T_{ij}\right). \end{array}$$

At present, in the business practice of enterprises, every enterprise manager is faced with a lot of jobs and challenges and there is no time and energy to deal with the risks that enterprises may face in the future. Therefore, if the risks are predicted and told to the managers of enterprises in advance, when making decisions, the investment in manpower capital will become easier and the possibility of risks will be less. The competition between enterprises is the competition of science and technology, and the carrier of science and technology is the employees of enterprises. If, for some reason, the core employees who master the technology of the enterprise jump to the competitive enterprise, while the investment cost of manpower capital is sunk, new manpower capital stock is added to the competitive enterprise and the enterprise will face more intense competition situation, which is extremely unfavorable to itself and affects the normal operation of the enterprise. Different risk levels reflect the degree of losses caused by manpower capital investment risks to enterprises, and different closed values can be set according to the risk levels of enterprises. One should warn and predict when it falls below this closed value, and when it exceeds this closed value, it means that the risk has become a reality.

## 4. Result Analysis and Discussion

When investing in manpower capital, enterprises should search for enough relevant information on the basis of investigation and research and make sufficient analysis and demonstration, so as to choose a reasonable investment scheme and reduce investment risks. The choice of investment objects of manpower capital in enterprises directly affects the whole process of investment in manpower capital. Excellent talents not only inject fresh blood into enterprises but also bring an efficient and positive working atmosphere to enterprises, which is of great significance to the long-term development of enterprises in the future. Analyzing the changing trends of the external environment, the national and government policies have a vital influence on the development direction of enterprises and enterprises should actively develop industries with policy support and relevant preferential measures. When making the outline of the strategic development plan of manpower capital investment, enterprises must stand at the height of long-term, sustained, and sustainable development and make a reasonable and comprehensive strategic plan of manpower capital, which conforms to the requirements of macro-manpower capital policies and the organizational structure of enterprises themselves and meets the needs of enterprises for manpower capital.

Ask experts to evaluate manpower capital investment projects and score their risks. According to the evaluation results of experts, from these three projects, the second project has the smallest risk, while the third project has the largest risk, as shown in Figure 3.

Due to various reasons, enterprises will have the demand for manpower capital investment; for example, due to the formulation of enterprise development strategy, the demand for manpower capital investment is caused by the difference between the existing talents of enterprises and expectations to a certain extent and the technological change of enterprises, which leads to the demand for manpower capital investment of enterprises for specific technical talents, and so on. Therefore, enterprises should be fully familiar with the internal manpower capital stock and development needs, understand their own manpower capital situation, and formulate enterprise manpower capital investment needs. The universal existence of individual differences in the rational allocation of personnel determines that everyone has his or her unique personality and each occupation has different requirements for various qualities of workers. Reasonable allocation of employees requires the matching of people and posts; that is, everyone is assigned to the most suitable position, and each position has the most suitable talents. This requires enterprises to fully understand each person's characteristics, advantages, and disadvantages, as well as the characteristics and job requirements of each post, and try their best to make the personal characteristics consistent with the professional environment.

Sensitivity analysis can be carried out for each influencing factor of a single project, and risk management can be carried out for the project from the analysis results. The relationship between risk evaluation and risk factor changes is shown in Figure 4.

The model is used to simulate the risk evaluation of manpower capital investment sample data, and the risk degree of the project is obtained. The comparison results are shown in Figure 5.

The simulation results are basically consistent with the recommended values given by experts, which shows that the model has high accuracy. When making the first demand plan of manpower capital, enterprises must fully consider two factors: market factors and their own manpower capital status. With the continuous growth and development of enterprises, the external environment is constantly changing and enterprises will have various talent needs. No matter what way to obtain these talents, enterprises must formulate reasonable manpower capital investment plans to serve enterprises. Enterprises need to timely introduce talents urgently needed by enterprises and timely promote qualified employees. At the same time, according to the work tasks, it can be determined whether employees require repetitive needs, short-term needs, or long-term needs. Through the establishment of a training effect training index and evaluation system, enterprises can check and evaluate whether the training has achieved the expected goal and whether the training plan is effective, so as to provide the basis for the next training plan and demand analysis. Because the investment object of manpower capital investment is a person with thought, individual behavior, and personality characteristics, it is different from the general investment object in complexity. Therefore, when investing in manpower capital, it is necessary to select suitable employees; otherwise, investing in the wrong object will increase the investment risk of the enterprise or even fail to recover the investment cost.

Sensitivity analysis can be made on the influencing factors of manpower capital investment projects, so as to analyze the effects of different factors on the projects. Take Project 2 as an example; if the influencing factors of benefit change by 5%, the risk early warning model based on data warehouse can be used to get the changed benefit evaluation value. The relationship between benefit evaluation and benefit influencing factors is shown in Figure 6.

After the completion of manpower capital investment, enterprises should first give timely evaluation feedback. In the process of putting manpower capital into use, enterprises should form a systematic manpower capital management mechanism. The development of employees' personality should not be ignored when establishing corporate culture and the common value of employees, because each employee has his own cognitive model, and only by respecting each employee can employees maximize their potential. After the investment is completed, the new manpower capital formed should be assessed, or an employee seminar can be held after the investment is completed to create a relaxed and happy conversation environment to ensure the value of this meeting. The content of the discussion mainly includes the feelings in the investment process, the harvest after the investment, the future work expectation, preliminary understanding of the gap between investment results and expectations, and so on. Employees in enterprises have the most contact with colleagues around them at work, and building good employee relations can effectively promote the enthusiasm of employees. Job analysis is the basis of job matching. Job analysis is to understand the tasks that should be completed in a certain job, their importance in the enterprise, and what qualifications employees should have to be qualified for this job.

Compare the relative importance of each factor in the same level with respect to the same factor in the previous level, and construct a pairwise comparison matrix. Invite experts engaged in manpower capital investment to evaluate and score indicators. Compare the indexes at the same level, and give the proportional scale score according to the relative importance of the indexes. After processing, the weight judgment matrix is constructed. The data relationship between weight and evaluation value is shown in Figures 7–9.

The evaluation of manpower capital investment projects is a key link to determine the success of investment operation. From the investor's point of view, enterprise value is a kind of benefit relationship between the satisfaction of investors' income needs and the satisfaction of investors' income needs. The evaluation of enterprise investment value follows the model and method of value evaluation.

After doing a good job analysis, we should grant corresponding authority according to the job responsibilities, distribute benefits reasonably, and formulate corresponding employee standards. Interpersonal relationships in organizations include the relationship between superiors and subordinates in working relationships, the relationship between leaders and members of organizations, the relationship between leaders, and the relationship between colleagues among members of organizations in the same position. Every member of an organization is in these two minimum relationships, and how these relationships are handled directly affects the organizational atmosphere, employee participation, and then organizational performance. The promotion of work needs different manpower capital to cooperate with each other, and it must be rationally allocated on the premise of understanding the nature of work and manpower capital. In a work team, each employee has different abilities and personalities, so it is necessary to define each employee's responsibilities and authority and create a good working atmosphere. In enterprises, we must establish the awareness of active communication and strengthen the communication between employees and between employees and superiors. Forming good interpersonal relationships in enterprises can reduce the internal transaction cost and reduce the investment risk of manpower capital.

## 5. Conclusions

With the advent of the information age, the contribution rate of knowledge to economic development has gradually increased and, accordingly, the competition among enterprises has changed from the competition of material resources to the competition of manpower capital. Therefore, it is an important part of enterprise's manpower capital investment risk management to reasonably assess the risks in the selection and use stages of manpower capital. Based on manpower capital theory, risk management theory, corporate governance theory, and risk early warning theory, this paper analyzes the characteristics of enterprise manpower capital investment risk, establishes a relatively perfect enterprise manpower capital investment risk early warning and control model, and analyzes relevant measures of risk prevention in order to reduce enterprise manpower capital investment risk. According to the formation process of manpower capital, manpower capital investment can be divided into recruitment and introduction investment, allocation and use investment, training investment, maintenance and establishment investment, and health protection investment. By establishing an integrated, efficient data warehouse with guaranteed data quality, the dependence on the business system database can be reduced. Integrating all kinds of information within the enterprise to make it tend to be consistent will not only reduce the operating cost of the enterprise but also enable customers to obtain consistent and complete information and services, ensure the information integration among various channels, and avoid the conflict of service content and caliber.

This paper lacks the dynamic analysis of manpower capital investment risk; that is, the time factor is brought into the theory of manpower capital investment, and the change of risk and its influence on the level of manpower capital investment due to the passage of time is specifically analyzed. The risk aversion system is only analyzed and studied theoretically and methodologically, without further verifying the scientificity and feasibility of the risk aversion system from the empirical point of view. In future research work, it is necessary to further standardize and improve the index system.

## Figures and Tables

**Figure 1:** Data warehouse system storage structure.

**Figure 2:** The functions of the enterprise manpower capital investment risk early warning system.

**Figure 3:** Technical risk data of risk evaluation results.

**Figure 4:** The relationship between risk assessment and changes in risk factors.

**Figure 5:** Comparison of recommended value and evaluation value data.

**Figure 6:** The relationship between benefit evaluation and benefit influencing factors.

**Figure 7:** Data relationship between the market environment risk weight value and evaluation value.

**Figure 8:** The relationship between the financial status risk weight value and the evaluation value data.

**Figure 9:** Data relationship between the customer risk weight value and evaluation value.

## Data Availability

The datasets used and/or analyzed during the current study are available from the corresponding author on reasonable request.

## References

[1] Schultz R. F., Sharathkumar A., Kwon S., Doerfer K., Lales G., Bhat R. (2020). Implementation of automatic data extraction from an enterprise database warehouse (EDW) for validating pediatric VTE decision rule: a prospective observational study in a critical care population. *Journal of Thrombosis and Thrombolysis*.

[2] Carson M. B., Scholtens D. M., Frailey C. N. (2016). Characterizing teamwork in cardiovascular care outcomes. *Circulation: Cardiovascular Quality and Outcomes*.

[3] Ranjan R (2016). Exploring inter-relationships among human-tiger conflicts, manpower capital outcomes for forest dependent communities and the sustainability of tiger habitats. *Human Ecology*.

[4] Duncan R., Toledo P. (2019). Inequality in body mass indices across countries: evidence from convergence tests. *Economics and Human Biology*.

[5] Handa S, Palermo T, Rosenberg M (2016). How does a national poverty programme influence sexual debut among Kenyan adolescents?. *Global Public Health*.

[6] King K. A. (2016). The talent deal and journey. *Employee Relations*.

[7] Montford W., Goldsmith R. E. (2016). How gender and financial self-efficacy influence investment risk taking. *International Journal of Consumer Studies*.

[8] Mijs J. J. B., Jonathan J. B. (2016). The unfulfillable promise of meritocracy: three lessons and their implications for justice in education. *Social Justice Research*.

[9] Ma A, Em B, So C (2019). Private equity and manpower capital risk. *Journal of Financial Economics*.

[10] Song S., Lee J. Y. (2017). Relationship with headquarters and divestments of foreign subsidiaries: the hysteresis perspective. *Management International Review*.

[11] Li S, Quan Y, Tian G. G, Kun T. W, Stella H. W (2021). Academy fellow independent directors and innovation. *Asia Pacific Journal of Management*.

[12] Uddin M. A., Ali M. H., Masih M. (2017). Political stability and growth: an application of dynamic GMM and quantile regression. *Economic Modelling*.

[13] Shir S (2018). Third Age under neoliberalism: from risky subjects to manpower capital.. *Journal of Aging Studies*.

[14] Israel S. (2016). More than cash: societal influences on the risk of material deprivation. *Social Indicators Research*.

[15] Martínez-Ferrero J., Banerjee S., García-Sánchez I. M. (2016). Corporate social responsibility as a strategic shield against costs of earnings management practices. *Journal of Business Ethics*.

[16] Schwager R., Eckwert B, Zilcha I (2016). Eckwert, Bernhard and Zilcha, Itzhak: the economics of screening and risk sharing in higher education: human capital formation, income inequality, and welfare. *Journal of Economics*.

[17] Hirst G., Walumbwa F., Aryee S., Butarbutar I., Chen C. J. H. (2016). A multi-level investigation of authentic leadership as an antecedent of helping behavior. *Journal of Business Ethics*.

[18] Shern D. L., Blanch A. K., Steverman S. M. (2016). Toxic stress, behavioral health, and the next major era in public health. *American Journal of Orthopsychiatry*.

[19] De Paola M., Gioia F. (2017). Does patience matter in marriage stability? Some evidence from Italy. *Review of Economics of the Household*.

[20] Caixe D. F., Kalatzis A. E. G., Castro L. R. K. d. (2019). Controlling shareholders and investment-risk sensitivity in an emerging economy. *Emerging Markets Review*.

[21] James B. E., Vaaler P. M. (2017). Experience, equity and foreign investment risk: a PIC perspective. *Management International Review*.

[22] Grant A., Satchell S. (2019). Endogenous divorce risk and investment. *Journal of Population Economics*.

[23] Chevalier A., Hirsch G. (2017). The assessment of the political risk in the investment decision. *Journal of the Operational Research Society*.

[24] Panteghini P. M., Vergalli S. (2016). Accelerated depreciation, default risk and investment decisions. *Journal of Economics*.

[25] King T., Loncan T., Khan Z. (2021). Investment, leverage and political risk: evidence from project-level FDI. *Journal of Corporate Finance*.

[26] Arora A., Gosain A. (2021). Intrusion detection system for data warehouse with second level authentication. *International Journal of Information Technology*.

